# The Effects of Target Skeletal Muscle Cells on Dorsal Root Ganglion Neuronal Outgrowth and Migration In Vitro

**DOI:** 10.1371/journal.pone.0052849

**Published:** 2013-01-14

**Authors:** Weiwei Zhang, Zhenzhong Li

**Affiliations:** Department of Anatomy, Shandong University School of Medicine, Jinan, China; Imperial College London, United Kingdom

## Abstract

Targets of neuronal innervations play a vital role in regulating the survival and differentiation of innervating neurotrophin-responsive neurons. During development, neurons extend axons to their targets, and then their survival become dependent on the trophic substances secreted by their target cells. Sensory endings were present on myoblasts, myotubes, and myofibers in all intrafusal bundles regardless of age. The interdependence of sensory neurons and skeletal muscle (SKM) cells during both embryonic development and the maintenance of the mature functional state has not been fully understood. In the present study, neuromuscular cocultures of organotypic dorsal root ganglion (DRG) explants and dissociate SKM cells were established. Using this culture system, the morphological relationship between DRG neurons and SKM cells, neurites growth and neuronal migration were investigated. The migrating neurons were determined by fluorescent labeling of microtubule-associated protein-2 (MAP-2) and neurofilament 200 (NF-200) or growth-associated protein 43 (GAP-43). The expression of NF-200 and GAP-43 and their mRNAs was evaluated by Western blot assay and real time-PCR analysis. The results reveal that DRG explants showed more dense neurites outgrowth in neuromuscular cocultures as compared with that in the culture of DRG explants alone. The number of total migrating neurons (the MAP-2-expressing neurons) and the percentage NF-200-immunoreactive (IR) and GAP-43-IR neurons increased significantly in the presence of SKM cells. The levels of NF-200 and GAP-43 and their mRNAs increased significantly in neuromuscular cocultures as compared with that in the culture of DRG explants alone. These results suggested that target SKM cells play an important role in regulating neuronal protein synthesis, promoting neuritis outgrowth and neuronal migration of DRG explants in vitro. These results not only provide new clues for a better understanding of the association of SKM cells with DRG sensory neurons during development, they may also have implications for axonal regeneration after nerve injury.

## Introduction

Targets of neuronal innervations play a vital role in regulation of the survival and differentiation of innervating neurotrophin (NT)-responsive neurons [1]. The motor neurons and skeletal muscle (SKM) fibers innervations depend on each other strongly [2]–[3]. Important communication between both tissues is mediated through the neuromuscular junction. Release and reception of various factors at other parts of both tissues must be considered as means of mutual influences [4]. Exchange of neurotrophins (NTs) and other molecules is likely to be an important source of nerve-muscle communication. NTs potentiate presynaptic release of neurotransmitter [5]–[6] and are essential for motor neuron survival [7], as well as for the maintenance of postsynaptic characteristic develop and maturation of muscle. Synapse-forming axons have vital effect on cell-surface behavior at nerve-muscle contacts during synaptogenesis in co-cultures of rat ventral spinal cord neurons and myotubes [8]. Neuromuscular junction development has been identified with co-cultures of dissociated embryonic neurons and SKM cells [9]. Innervations induce formation of a mature SKM-like excitation-contraction coupling system in cultured human muscle cells [10]. Peripheral nerve recovery after crush injury was suppressed by chronic inflammation in peripheral target tissue [11]. Extracellular application of myosin II or skeletal muscle extract to neurons resulted in a robust increase in the number of axons initiated by each neuron or the number of survival neurons [12]–[13]. Sensory nerve cross-anastomosis (sensory protection) provides a modified trophic environment by modulating neurotrophic factor synthesis in muscle [14].

Microtubule associated protein-2 (MAP-2), which is very abundant in the mammalian nervous system, has been associated with the formation of neurites at early developmental stages and with the dendrite scaffold upon maturation [15]. MAP-2 has been used as a sensitive and specific marker for neurons [16]. Neurofilaments (NFs) are neuron-specific intermediate filaments. They are classed into three groups according to their molecular masses: neurofilament heavy, middle and light chains (NF-H, NF-M and NF-L). They maintain and regulate neuronal cytoskeletal plasticity through the regulation of neurites outgrowth, axonal caliber and axonal transport [17]. NF-H plays an important role in healthy neurons [18].

Growth-associated protein-43 (GAP-43), an axonally localized neuronal protein, plays a major role in many aspects of neuronal function in vertebrates [19]–[20]. GAP-43 may express in all subpopulations of small and large dorsal root ganglion (DRG) neurons [21]–[22] and plays an important role in growth cone formation and neurites outgrowth of cultured DRG neurons [23]. GAP-43 is an intracellular growth-associated protein that appears to assist neuronal pathfinding and branching during development and regeneration [24]. Increases of GAP-43 are a frequently used marker of nerve regeneration or active sprouting of axons after traumatic injury in vivo [25]–[29] and an indicator of neuronal survival in vitro [30]–[31].

The knowledge of mutual interactions between postsynaptic receptors and presynaptic partner neurons during development and differentiation is very limited [32]. New interpretations of prior knowledge between neurons and muscle cells have been promoted by the preparations of the neuromuscular cocultures of motor neurons and SKM cells [33]. The interdependence of sensory neurons and SKM cells during both embryonic development and the maintenance of the mature functional state had not been fully understood. We hypothesized that target SKM cells may promote neuronal outgrowth, migration and expression of neuronal proteins. In the present study, neuromuscular cocultures of organotypic DRG and SKM cells were established. Using this culture system, we investigated the contribution of target tissues to neuronal outgrowth, migration and expression of neurofilament 200 (NF-200) and GAP-43.

## Results

### Morphology of DRG neurons and SKM cells in neuromuscular cocultures

In the DRG explants cultures, the DRG explants sent large radial projections to the peripheral area. The axons formed a lace-like network with crossing patterns in the peripheral area. The single migrating neurons scattered in the space of the network and sent axons to join the network (Fig. 1).

**Figure 1:** SEM photomicrographs of the neuromuscular coculture (A–F) and DRG explants culture alone (G–I). Panel A: DRG explants send numerous large radial projections (thin arrows) to the peripheral area in neuromuscular coculture. Many neurons (thick arrows) migrated from DRG explants to the peripheral area. Panel B: The enlargement of the box in Panel A. Panel C: The axons form a dense lace-like network (thin white arrows) with crossing patterns on the surface of single layer SKM cells (thick black arrow) in neuromuscular coculture. The single migrating neurons (thick white arrows) scattered in the space of the network and send axons (thin black arrows) joining the network. Panel D: The axons cross (thin white arrows) on the surface of a single SKM cell (thick black arrow). Panel E: The endings of the axons enlarge and terminate on the surface of a single SKM cell (thick black arrow) to form NMJ-like structures (thin white arrows). Panel F: The enlargement of the box in Panel E. Panel G: DRG explants sends radial projections (thin arrows) to peripheral area in DRG explants culture. A few neurons (thick arrows) migrated from DRG explants to the peripheral area. Panel H: The enlargement of the box in Panel G. Panel I: The axons form a sparse lace-like network (thin white arrows) with crossing patterns in the peripheral area in DRG explants culture. The single migrating neuron (thick white arrow) sends axons (thin black arrow) joining the network. Scale bar = 50 µm in Panel A, G; Scale bar = 25 µm in Panel B, H; Scale bar = 10 µm in Panel C; Scale bar = 5 µm in Panel D, E, I; Scale bar = 2.5 µm in Panel F.

In neuromuscular coculture, most of SKM cells are fused to form myotubes which maybe branched or take the shape of long rods. The axons from DRG explant frequently. Some axons terminate upon contact with the contracting SKM cells, others may choose to ignore the surfaces of SKM cells. The axons would cross each other to form a fine network on the surface of the single layered SKM cells. The crossing axons adhere to each other hence the displacement of one terminal axon on a contracting muscle cell would also oscillate the proximally area of the axonal network. The configurations of the terminal axons observed under SEM were variable. Some axons would widen into a varicosity, some would become smaller in caliber and many others appear to be no different from the immediate proximal configuration. The endings enlarge and terminate on the surface of SKM cells to form neuromuscular junction (NMJ)-like structures (Fig. 1,2).

**Figure 2:** Double fluorescent labeling of MAP-2 (for neurons) and muscle actin (for muscle cells). Panel A : MAP-2 for DRG neurons; Panel B: muscle actin for SKM cells; Panel C: overlay of Panel A and B. The migrating neurons send axons cross over (thick arrow) and terminate on (thin arrow) the surface of SKM cells. Scale bar = 50 µm.

### The number of nerve fiber bundles extended from DRG explants

At 6 days of culture age, DRG explants sends large radial projections 5∼15 µm in diameter to peripheral area. The number of nerve fiber bundles in neuromuscular coculture of DRG explants and SKM cells is 20.80±1.91. The number of nerve fiber bundles in DRG explants culture is 6.90±0.86. The number of nerve fiber bundles increased very significantly in the presence of target SKM cells (*P*<0.001) (Fig. 3).

**Figure 3:** Nerve fiber bundles extended from DRG explants. Panel A, B: The example images to show how to quantify nerve fiber bundles. Nerve fiber bundles extended from DRG explants as far as 200 µm from the edge of a quarter of each DRG explants was counted in each sample. Panel A is neuromuscular coculture (thick arrows show SKM cells). Panel B is DRG explant culture. Panel C: The number of nerve fiber bundles extended from DRG explants. The number of nerve fiber bundles increased in neuromuscular coculture as compared with that in DRG explants culture alone. Bar graphs with error bars represent mean ± SEM (n = 10 different samples). *P<0.001. Scale bar = 40 µm.

### Total migrating neurons from DRG explants

Neuron migration from DRG explants begins 24 hours after plating. After 2 days, the individual neurons migrate from DRG explants to peripheral area. After 6 days, more and more individual neurons migrate from DRG explants. The migration distance can be up to several hundred micrometers into the peripheral area around the explants. These individual neurons were multipolar or bipolar in configuration with central bodies up to 15 by 40 µm in size. The total number of neurons migrated from DRG explants in neuromuscular cocultures is 35.29±1.65. The total number of migrating neurons in DRG explants culture alone is 16.61±1.16. The presence of target SKM cells promoted neuronal migration form DRG explants in the neuromuscular cocultures (*P*<0.001) (Fig. 4,5).

**Figure 4:** The example images to show how to count cells. The full visual field showed in the circle in which neurons were counted in one sample. The neurons in the box were showed in figure 6. Panel A is the total neurons (MAP-2-IR neurons). Panel B is NF-200-IR neurons. Panel C is the overlay of Panel A and B.

**Figure 5:** Total migrating neurons from DRG explants. Total number of migrating neurons from DRG explants increased in neuromuscular coculture as compared with that in DRG explants culture alone. Bar graphs with error bars represent mean ± SEM (n = 38 different samples). *P<0.001.

### The percentage of NF-200-IR neurons and GAP-43-IR neurons

To test the effects of SKM cells on NF-200 and GAP-43 expression in migrating DRG neurons from DRG explants, cultures of DRG explants were incubated for 6 days in the presence or absence of SKM cells and processed for double fluorescent labeling of MAP-2 and NF-200 or GAP-43, and then the percentage of DRG neurons containing NF-200 or GAP-43 was quantified. The percentage of NF-200-IR (54.78%±3.89%) migrating neurons from DRG explants in neuromuscular cocultures is higher than that in DRG explants culture alone (41.34%±3.25%) (*P*<0.05) (Fig. 6). The percentage of GAP-43-IR (76.59%±1.49%) migrating neurons from DRG explants in neuromuscular coculture is also higher than that in DRG explants culture alone (39.86%±2.10%) (*P*<0.001) (Fig. 7).

**Figure 6:** Double fluorescent labeling of MAP-2 and NF-200. Panel A: neuromuscular coculture (A1: MAP-2; A2: NF-200; A3: overlay of A1 and A2). Panel B: DRG explant culture (B1: MAP-2; B2: NF-200; B3: overlay of B1 and B2). Panel C: The percentage of migrating NF-200-IR neurons. The percentage of NF-200-IR neurons increased in neuromuscular coculture as compared with that in DRG explants culture alone. Bar graphs with error bars represent mean ± SEM (n = 20 different samples), Scale bar = 50 µm. *P<0.05.

**Figure 7:** Double fluorescent labeling of MAP-2 and GAP-43. Panel A: neuromuscular coculture (A1: MAP-2; A2: GAP-43; A3: overlay of A1 and A2). Panel B: DRG explant culture (B1: MAP-2; B2: GAP-43; B3: overlay of B1 and B2). Panel C: The percentage of migrating GAP-43-IR neurons. The percentage of GAP-43-IR neurons increased in neuromuscular coculture as compared with that in DRG explants culture alone. Bar graphs with error bars represent mean ± SEM (n = 18 different samples), Scale bar = 50 µm. *P<0.001.

### The mRNA levels of NF-200 and GAP-43

To determine the mRNA levels of NF-200 and GAP-43, the DRG explants at 6 days of culture age in the presence or absence of SKM cells were analyzed by real time-PCR. NF-200 mRNA levels increased in neuromuscular cocultures (1.75±0.09 folds, *P*<0.001) as compared with that in DRG explants culture alone. Similarly, GAP-43 mRNA levels also increased in neuromuscular cocultures (2.00±0.16 folds, *P*<0.01) as compared with that in DRG explants culture alone (Fig. 8).

**Figure 8:** The mRNA levels of NF-200 and GAP-43. The mRNA levels of NF-200 and GAP-43 increased in neuromuscular coculture as compared with that in DRG explants culture alone. Bar graphs with error bars represent mean ± SEM (n = 6). *P<0.01, **P<0.001.

### The protein levels of NF-200 and GAP-43

To determine the protein levels of NF-200 and GAP-43, the DRG explants at 6 days of culture age in the presence or absence of SKM cells were analyzed by Western blot assay. NF-200 protein levels increased in neuromuscular cocultures (1.46±0.02 folds, *P*<0.001) as compared with that in DRG explants culture alone (Fig. 9). GAP-43 protein levels increased in neuromuscular cocultures (1.68±0.04 folds, *P*<0.001) as compared with that in DRG explants culture alone, too (Fig. 10).

**Figure 9:** The protein levels of NF-200. The protein levels of NF-200 increased in neuromuscular coculture as compared with that in DRG explants culture alone. Bar graphs with error bars represent mean ± SEM (n = 6). *P<0.001.

**Figure 10:** The protein levels of GAP-43. The protein levels of GAP-43 increased in neuromuscular coculture as compared with that in DRG explants culture alone. Bar graphs with error bars represent mean ± SEM (n = 6). *P<0.001.

## Discussion

During development, neurons extend axons to their targets. The neurites' survival then becomes dependent on the trophic substances secreted by their target cells [34]. Target tissues contribute to the phenotypic and functional development of sensory neurons [35]–[36]. The interdependence of sensory neurons and SKM cells has not been fully understood. To better understand the interactions between sensory neurons and SKM cells, neuromuscular cocultures of organotypic DRG explants and dissociate SKM cells were established in the present study. Using this culture system, the morphological relationship between DRG neurons and SKM cells, neurites growth and neuronal migration were investigated. The results reveal that DRG explants show denser neurites outgrowth in neuromuscular cocultures as compared with that in the culture of DRG explants alone. The number of total migrating neurons (the MAP-2-expressing neurons) and the percentage of NF-200-IR and GAP-43-IR neurons increased significantly in the presence of SKM cells. Furthermore, the levels of NF-200 and GAP-43 and their mRNAs also increased significantly in neuromuscular cocultures as compared with that in the culture of DRG explants alone. These results suggested that target SKM cells play an important role in the regulation of neuronal protein synthesis, promoting neurites outgrowth and neuronal migration of DRG explants in vitro.

MAP-2 is a cytoskeletal protein. It plays a regulatory role in neuronal plasticity and in maintaining the morphology of differentiated neurons [37]. MAP-2 has been tentatively implicated in neuronal outgrowth and polarity of neuronal cells [15]. It has been shown that MAP-2 is specifically expressed in neuronally differentiated cells [16]. MAP-2 is a cytoskeletal phosphoprotein that regulates the dynamic assembly characteristics of microtubules and it appears to provide scaffolding for organelle distribution into the dendrites and for the localization of signal transduction apparatus in dendrites [38]. It has been suggested that MAP-2 can interact with cytoskeletal components and might be critically involved in neurites initiation [39]. Within the neuronal cell, MAP-2 proteins are known to interact with β-tubulin, neurofilaments (NFs) and actins, and contribute to dendrite outgrowth and maintenance of neuronal cytoarchitecture [40]–[41]. In the present study, MAP-2 was used as a neuronal marker to detect neurons in different culture conditions. The migrating MAP-2-IR neurons increased significantly in neuromuscular cocultures as compared with that in DRG cultures. These results suggested that target SKM cells' participation in regulating DRG neuronal migration in vitro is fundamental.

The number of neurons migrated from DRG explants and the number of nerve fiber bundles extended from DRG explants represent the outgrowth state of organotypic DRG explants in cultures. In the present study, we also observed that the number of nerve fiber bundles increased significantly in neuromuscular coculture as compared with that in DRG culture alone. These results suggested that target SKM cells play a very important role in regulating DRG neuronal neurites outgrowth and maintenance of neuronal cytoarchitecture in vitro. Interestingly, this in vitro model indicates that the primary sensory nerve endings and SKM cells are much more closely related morphologically than those in vivo conditions. The present study provides novel evidence that the formation of NMJ-like structures may exist in the co-culture of organotypic DRG neurons and SKM cells. This result implicated that anatomical neuromuscular contact between sensory neurons and SKM cells, or the morphological sensory innervations of dissociated SKM cells was established in vitro. Once neurons recognize their appropriate targets, specific neuron-target contacts will be established. These contacts are involved with modulation of neurites growth dynamics and the formation of functional synaptic connections [42]–[44]. Cell-cell recognition often requires the formation of a highly organized pattern of receptor proteins in the intercellular junction, like a synapse [45]. The mechanisms of the formation of NMJ-like structures observed in the present experiment may depend on the different proteins synthesized in both DRG neuronal terminals and target SKM cells.

NF-H (NF-200) plays an important role in healthy neurons [18]. The appearance of NF-H represents a critical event in the stabilization of axons that accompanies their maturation [46]. In the present study, the percentage of NF-200-IR neurons, NF-200 protein and its mRNA expression ratio increased significantly in the presence of target SKM cells. These results suggested that target SKM cells are important not only for promoting NF-200-IR neuronal migration but also for maintaining NF-IR neuronal phenotype.

GAP-43 is a membrane-bound molecule expressed in neurons. It is particularly abundant during periods of axonal outgrowth in development and regeneration of the central and peripheral nervous systems. It is known that GAP-43 mRNA is expressed in the DRG of adult rat and that GAP-43 is upregulated in DRG neurons during regeneration [47]. The expression of GAP-43 mRNA is higher in DRG neurons after peripheral nerve lesions [48]. A recent study has shown that the enhancement of neurites outgrowth is associated with the expression of GAP-43 in DRG cultures [49]. The expression of GAP-43 mRNA in primary cultured DRG neurons correlates very well with morphological changes of neurites degeneration [50]. The enhanced growth state is accompanied by an increase in the expression of GAP-43 in preinjured but not intact DRG [51]. In the present study, organotypic cultured DRG explants seem to represent an injured state, since the neurons are axotomized during culture preparation. In this experiment, the percentage of GAP-43-IR neurons, the levels of GAP-43 protein increased parallelly with its mRNA in the neuromuscular cocultures as compared with that in the culture of DRG explants alone. These results suggested that target SKM cells play an important role in neurites regeneration from DRG explants in vitro.

The percentage of NF-200-IR and GAP-43-IR neurons as well as the number of total migrating neurons (the MAP-2-expressing neurons) increased significantly in the presence of target SKM cells suggested that target SKM cells not only promoted neuronal migration but also promoted neurite regeneration and maintained NF-IR neuronal phenotype which might contact with muscle spindle [52]. The formation of NMJ-like structures between enlarged nerve endings and the surface of SKM cells observed in the present study suggesting more closely relationship between the neurites and muscle cells in vitro as compared with that happened in vivo. Hence, the results of the present study provide new insights for further exploring the mutual interactions between postsynaptic receptors and presynaptic partner neurons during development and differentiation.

In conclusion, the results of the present study suggested that target SKM cells play an important role in regulating neuronal protein synthesis, maintaining neuronal survival and plasticity, promoting neurites outgrowth and neuronal migration of DRG explants in vitro. These results not only provide new clues for a better understanding of the association of target SKM cells with DRG sensory neurons during development, but they also show the target SKM cells may have implications for axonal regeneration after nerve injury.

## Materials and Methods

### Ethics Statement

All animals were cared for in accordance with the National Institute of Health Guide for the Care and Use of Laboratory Animals (revised 1996; http://www.nap.edu). All procedures described herein were reviewed by and had prior approval by the Ethical Committee for Animal Experimentation of the Shandong University. All surgery was performed under anesthesia, and all efforts were made to minimize suffering of the animals.

### Cell culture preparations

The organotypic DRG culture preparations utilized embryonic rats taken from the breeding colony of Wistar rats maintained in the Experimental Animal Center at Shandong University of China. DRG explants were obtained from embryonic day 15 (E15) rat embryos. Under aseptic conditions, the bilateral dorsal root ganglia (DRGs) were removed from each rat embryo by microforceps and placed in culture media in half of Petri dishes and used for neuromuscular cocultures. Each DRG explants was plated at the bottom of each well of 24-well clusters (Costar, Corning, NY, USA).

SKM cell culture preparations utilize newborn Wistar rats. SKM cell cultures were prepared 3 days prior to DRG preparation. In brief, limbs of neonatal rats were collected in Ca^2+^ and Mg^2+^ -free Hanks' balanced salt solution on ice. Muscles were removed and cut into fragments approximately 0.5 mm in diameter, After digestion with 0.25% trypsin (Sigma, USA) in D-Hanks solution at 37°C for 40 minutes, the cell suspension was filtered through 200 molybdenum copper mesh, centrifuged, and triturated in growth media supplemented with 5% fetal bovine serum (Gibco, Origin: Australia). Isolated SKM cells were plated at a density of 2×10^5^ cells/ml in 24-well clusters (Costar, Corning, NY, USA) which would contain 24 mm diameter coverslips precoated with poly-L-lysine (0.1 mg/ml). The 24-well clusters culture dish is then placed in incubator with proper culture environment, 37°C and 5% CO_2_.

The neuromuscular coculture is prepared as following: Each newly prepared DRG explants was plated into a well with 3-day old SKM culture after confluency myoblast fusion has happened. The coculture with SKM cells is allowed to grow for an additional 6 days with media change every 2 days.

The composition of the culture media is DMEM/F-12 (1∶1) supplemented with 10% fetal bovine serum (Gibco, Origin: Australia), 2% B-27 supplement (Gibco, Grand Island NY, USA), L-glutamine (0.1 mg/ml, Sigma, USA), insulin (0.25 µg/ml), penicillin (100 U/ml), and streptomycin (100 µg/ml).

### Observation of morphological relationship between DRG neurons and SKM cells

At 6 days of culture age, DRG cultures and neuromuscular co-culture were processed for scanning electron microscopy (SEM) examination. The samples were rinsed quickly once in 0.01 mol/L PBS and prefixed in 2.5% glutaraldehyde solution for 12 hours. Post-fixation was done with a 1% osmium tetroxide solution for 90 minutes. After dehydrated in graded ethanol, the samples were treated with dehydrated alcohol/acetone solution (1∶1) for 20 minutes, acetone for 30 minutes, and acetone/camphene solution (1∶1) for 30 minutes, respectively. Then the samples were treated with liquid camphene twice for 20 minutes each at 45°C. After vacuum drying, the samples were covered with platinum by ion sputtering and examined under SEM (Hitachi S-570).

### Determination of neurites outgrowth from DRG explants

At 6 days of culture age, the number of nerve fiber bundles extended from DRG explants both in DRG culture alone or neuromuscular coculture was counted. Nerve fiber bundles extended from DRG explants as far as 200 µm from the edge of a quarter of each DRG explants was counted in each sample. The length of nerve fiber bundle which is less than 200 µm was not counted in this experiment.

### Immunocytochemistry

At 6 days of coculture age, DRG cultures and neuromuscular coculture were processed for immunofluorescent labeling. The cultures were rinsed quickly once in 0.1 mol/L phosphate buffer saline (PBS) to remove medium. The cells were fixed in 4% paraformaldehyde, pH 7.4, for 40 minutes at 4°C. After washing in 0.1 mol/L PBS for 3 times, the cells were blocked by 10% normal goat serum after 0.6% Triton X-100 PBS to block non-specific sites and permeabilize cells. The samples were incubated with primary antibody overnight at 4°C. After washing in 0.1 mol/L PBS 3 times, the samples were incubated by second antibody for 60 minutes in dark at 37°C. After washing 3 times in 0.1 mol/L PBS, the cells were coverslipped immediately with Vectashield anti-fade mounting media (Santa Cruz Biotechnology, USA) and stored at 4°C until observation by fluorescent microscope.

Primary antibody: mouse monoclonal anti-MAP-2 (1∶400, abcam, Hong Kong); rabbit polyclonal anti-NF200 (1∶500, abcam, Hong Kong); rabbit monoclonal anti-GAP-43 (1∶1,000, abcam, Hong Kong); rabbit polyclonal anti-muscle actin (1∶500, Abcam, Hong Kong). Second antibody: goat anti-mouse conjugated to Cy2 (1∶400, abcam, Cambridge, UK); goat anti-rabbit conjugated to Cy3 (1∶400, abcam, Cambridge, UK).

### Determination of total migrating neurons and the percentage of NF-200-IR or GAP-43-IR neurons from DRG explants

Total migrating neurons from DRG explants were determined as MAP-2-immunoreactive (IR) neurons under a fluorescence microscopy (Olympus) with 20× objective lens. MAP-2-IR neurons in one visual field at the edge of DRG explants were counted as the total migrating neurons in each sample.

The migrating NF-200-IR or GAP-43-IR neurons from DRG explants were observed under a fluorescence microscope (Olympus) with 20× objective lens. NF-200-IR or GAP-43-IR neurons in one visual field at the edge of DRG explants were counted as the migrating NF-200-IR neurons in each sample. The numbers of total neurons (MAP-2-IR neurons) were also counted in the same visual field. Then, the percentage of NF-200-IR or GAP-43-IR neurons could be obtained.

### Real time-PCR analysis of mRNAs for NF-200 and GAP-43

The mRNA levels of NF-200 and GAP-43 in neuromuscular co-culture and DRG culture alone at 6 days of culture age were analyzed by real time-PCR analysis. The DRG explants were removed from 24-well clusters by microforceps. The expression of glyceraldehyde-3-phosphate dehydrogenase (GAPDH) mRNA was also determined as an internal control. Total DRG RNA was isolated by TRIzol (TakaRa, Japan). cDNA was synthesized using cDNA synthesis kit (Fermentas, Canada) according to the manufacturer's instructions, followed by PCR amplification.

Specific primers were used together with SYBR green to assess expression levels according to the manufacture's instructions. PCR were performed at 50°C for 2 minutes, 94°C for 15 minutes, followed by 40 cycles at 94°C for 15 seconds, 58°C for 30 seconds, and 72°C for 30 seconds.

In all cases, data were normalized for any minor variations in expression level of the housekeeping gene GAPDH. Data were expressed as fold induction using the 2^-ΔΔCt^ method. Primer sequences for each gene examined are shown as follow: NF-200 5′- AAA GTG AAC ACG GAT GCT ATG C -3′ (coding sense) and 5′- GTG CTT TTC AGT GCC TCC AAC -3′ (coding antisense). GAP-43 5′- AAG AAG GAG GGA GAT GGC TCT -3′ (coding sense) and 5′- GAG GAC GGC GAG TTA TCA GTG -3′ (coding antisense). GAPDH 5′- GGC ACA GTC AAG GCT GAG AAT G -3′ (coding sense) and 5′- ATG GTG GTG AAG ACG CCA GTA -3′ (coding antisense).

### Western blot assay of NF-200 and GAP-43 protein

The protein levels of NF-200 and GAP-43 in DRG in neuromuscular coculture and DRG culture alone at 6 days of culture age were analyzed by Western blot assay, with β-actin as an internal control. The DRG explants were removed from 24-well clusters on ice and homogenized in 10 mmol/L Tris homogenization buffer (pH 7.4) with protease inhibitors (Sigma, USA). The samples were centrifuged at 10,000 g for 20 minutes at 4°C. After determining the protein concentrations of the supernatants (BCA method, standard: BSA), about 50 µg protein per lane were resolved by SDS-PAGE (10%), and telectrotransferred to nitrocellulose membranes followed by blocking with 5% dry milk powder for 1 h and immunostaining with the respective primary antibody dilution for 1 to 4 h at RT or over night at 4°C. The membranes were incubated with primary antibodies: rabbit anti-NF-200 polyclonal IgG (1∶1,000, abcam, Hong Kong); rabbit anti-GAP-43 monoclonal IgG (1∶100,000, abcam, Hong Kong); or mouse anti-β-actin monoclonal IgG (1∶4,000, Santa Cruz Biotechnology, USA). After being washed three times for 10 minutes with washing solution, the membranes were incubated with second antibody: goat anti-rabbit IgG-HRP (1∶5,000, Santa Cruz Biotechnology, USA) or goat anti-mouse IgG-HRP (1∶4,000, Santa Cruz Biotechnology, USA). Peroxidase activity was visualized with the ECL Western blotting detection kit (Millipore, Billerica, USA) according to the manufacturer's instructions, and protein content was determined by densitometrically scanning the exposed x-ray film and the images were analyzed quantitatively by using an *ImageJ* 1.39u image analysis software. The levels of NF-200 and GAP-43 were expressed as the ratio of the protein to β-actin.

### Statistical analysis

Data are expressed as mean ± SEM. All the data were processed for verifying normality test for Variable. The normality tests have passed for all the data. Statistical analysis was evaluated with SPSS and GraphPad Prism 5.0 statistical software by *t* test for analysis of two independent samples. Significance was determined as *P*<0.05.
